The article "A Novel Sentiment Analysis Model of Museum User Experience Evaluation Data Based on Unbalanced Data Analysis Technology" was published in 2022. Journal: Comput Intell Neurosci.

# A Novel Sentiment Analysis Model of Museum User Experience Evaluation Data Based on Unbalanced Data Analysis Technology

**DOI:** 10.1155/2022/2096634

**Published:** 2022-04-28

**Authors:** Xiang Chen, Zhiwei Chen, Lei Xiao, Ming Zhou

**Affiliations:** ^1^School of Design, Jiangnan University, Jiangsu, Wuxi 214122, China; ^2^Graduate School Design, Dongseo University, Jurye-Ro, Busan 47011, Republic of Korea

## Abstract

With the development of virtual reality and digital reconstruction technology, digital museums have been widely promoted in various cities. Digital museums offer new ways to display and disseminate cultural heritage. It allows remote users to autonomously browse displays in a physical museum environment in a digital space. It is also possible to reproduce the lost heritage through digital reconstruction and restoration, so as to digitally present tangible cultural heritage and intangible cultural heritage to the public. However, the user's experience of using digital museums has not been fully and deeply studied at present. In this study, the user's experience evaluation data of digital museum are classified and processed, so as to analyze the user's emotional trend towards the museum. Considering that the user's evaluation data are unbalanced data, this study uses an unbalanced support vector machine (USVM) in the classification of user evaluation data. The main idea of this method is that the boundary of the support vector is continuously shifted to the majority class by repeatedly oversampling some support vectors until the real support vector samples are found. The experimental results show that the classification obtained by the used USVM has a good practical reference value. Based on the classification results of the evaluation data, the construction of the digital museum can be further guided and maintained, thereby improving the user experience satisfaction of the museum. This research will make an important contribution to the construction of the museum and the inheritance of culture.

## 1. Introduction

Museums play the role of cultural dissemination and entertainment in people's daily life and are deeply loved by the masses. However, traditional museums are limited in time and space, and their exhibition methods and contents are relatively simple. In addition, in order to watch the intangible cultural heritage exhibition, people need to go to the exhibition location to watch it, which will increase the cost of transportation, accommodation, and time, making people discouraged. In the era of information technology development, the development and application of virtual reality technology provide a new way to solve the above dilemma. The digital museum built with virtual reality technology has impacted the inherent existing form and static display mode of cultural relics. Through digital image rendering and animation technology, the original appearance of the museum can be reproduced. Digital museums allow people to walk into the museum without leaving their homes, with an immersive feeling. This method greatly reduces the time and capital costs for both the museum and the audience. Digital museums have become a direction that museums have been working on in recent years, with very broad prospects for development. The further development of digital museums in the future not only needs to consider user-centered construction issues but also needs to consider the effectiveness of cultural information dissemination. Therefore, establishing a reasonable and complete user experience evaluation system is an important research direction for digital museums. At present, most of the research on digital museums focus on two aspects. One is the research on the construction and management of digital museums. The other is the research on the dissemination methods, channels, and dissemination effects of cultural information in digital museums. These two research complement each other and influence each other. The quality of digital museum construction will affect the way and effect of its dissemination. The user's experience of the museum can guide the optimization of the museum construction.

At present, the construction of digital museum mainly has the following problems: first, the advantages of digital technology are not fully utilized, and the content of digital museums remains consistent with traditional museums. Second, the visual design of the user interface is simple and lacks aesthetic and cultural implications. Third, the operation is not smooth due to technical reasons. In order to improve the user experience of virtual exhibition halls, scholars at home and abroad have conducted many studies. Reference [1] evaluated the experience of three groups of children when using virtual exhibition halls to teach children in schools. The research shows that exhibition areas, remote lectures by museum staff, and interaction with children are all integral to virtual exhibitions. Reference [2] develops a Java program of personalized virtual exhibition tour based on World Wide Web thinking, to test whether the communication and cooperation between users can enhance the user's interest in use. Reference [3] explores how to improve interactive behaviors to enhance the user experience by studying user feedback on the “Keys To Rome” interactive virtual exhibition. Reference [4] introduces user experience into the research of virtual exhibition platform and puts forward the relevant theories of virtual exhibition platform research based on user experience through eye-tracking experiments and user survey research. Reference [5] discusses the realization of user experience model and virtual exhibition prototype system based on a computer multimedia environment. Reference [6] proposes to interpret traditional Chinese paintings with commentary dubbing and ambient sound to enhance user experience. When the user watches Chinese paintings, the system can judge the user's position and viewing direction according to the user's actions and visual center points, so as to synthesize stereo sound and play it.

Based on the above research, it can be analyzed that the determination of the user experience evaluation model is very important. The researchers designed questionnaires according to the research content and processed the collected data, using NASA-TLX scale [7], SWAT scale [8], factor analysis method [9], principal component analysis method [10, 11], and analytic hierarchy process [12] to build a quantitative model of user experience. Reference [13] points out that the construction of user experience model is the basis for evaluating user experience and divides the model into two types: structural model and measurement model. Reference [14] proposes a structural model of user engagement. It analyzes six attributes of engagement through validity and exploration factors, namely, perceived usability, aesthetics, attention span, sensory relevance, innovation, and persistence and through the structural equation model to determine the relationship between the various properties. Reference [15] established a total of five evaluation models: the traditional user satisfaction model, the usability research linear evaluation model, the linear model, the S-value model, the joint model, and the disjunctive model. In order to optimize the construction of the museum and improve the user's somatosensory experience, this study first designs a user questionnaire to collect user evaluation data. Second, considering that in the evaluation data, negative evaluations generally account for a small amount of the total data, so there will be a large gap in the magnitude of the two categories. Traditional classification methods are not competent for the classification of such data. This study introduces an imbalanced data processing method. For the collected and preprocessed data, this study uses the USVM algorithm to apply the sentiment classification of user evaluation data. Finally, based on the evaluation results obtained from the experimental analysis, the construction and optimization of the digital museum are guided.

### 1.1. Sentiment Classification Theory Model USVM

Various intelligent algorithms are often used in emotion analysis and other fields [16–18]. The core idea of used USVM is as follows: first, the original unbalanced data are divided into three areas: support vector area (SV), majority class nonsupport vector area (MNSV), and minority class nonsupport vector area (FNSV) according to the location. Second, the samples in the MNSV area and the FNSV area are denoised. Third, the oversampling process is repeated for a small number of samples that are misclassified in the SV area and partially correctly classified close to the decision boundary, until the training data set with the best test results is found. Finally, some samples in the MNSV area are randomly deleted.

When using the support vector machine (SVM) to classify unbalanced data, the interference of noise and the lack of true support vectors of minority classes are the main reasons for the poor classification effect of SVM on unbalanced data. Therefore, it is very necessary to remove noise samples and increase a few real support vector samples after classification. At the same time, in order to avoid the influence of sample differences between classes on the classification results as much as possible, it is necessary to selectively delete some majority class samples. The specific operation steps of each link are described as follows:

#### 1.1.1. Denoising

When using SVM to classify unbalanced data, since the decision boundary will shift to the side with fewer samples, the noise samples located in the MNSV area are not necessarily real noise samples. In order to identify all the noisy samples in the MNSV region, it is necessary to obtain k-nearest neighbors for all the minority class samples located in the MNSV region. If none of the *k* samples belong to the minority class, it is considered as noise. The steps of denoising are as follows:

#### 1.1.2. Oversampling the Samples in the FNSV Area

When classifying unbalanced data, the decision boundary of the classifier will be skewed, so that the obtained support vector samples are not necessarily all real support vector samples. Therefore, in order to obtain the most realistic support vector samples, it is necessary to repeat the oversampling process for the SV-classified misclassified samples and the minority class samples that are correctly classified and close to the decision boundary. The oversampling steps are as follows:

#### 1.1.3. Undersampling the Samples in the MNSV Area

Since samples in different positions may have different effects on the results of the classifier, it is unreasonable that the difference between samples between classes only refers to the difference in the number of samples. In comparison, it is reasonable that the difference between the accuracy of the minority class and the majority class test sample is the difference between the samples. The steps of undersampling are as follows:

The execution flow of the USVM algorithm is shown in Figure 1

## 2. User Experience Sentiment Classification Based on USVM

### 2.1. Experimental Data and Evaluation Indicators

In order to verify the performance of the sentiment classification model used in this study as objectively and accurately as possible, this study first uses public datasets to conduct experiments. This study selects two datasets of SemEval 2014 task 4, both of which are English datasets. SemEval 2014 task 4 includes the Restaurant review dataset and Laptop review dataset, which are divided into the training set and test set. Both training set and test set contain positive, neutral, and negative sentiment polarities, which are respectively 1, 0, and −1. The descriptions of the two datasets are listed in Table 1.

The evaluation indicators used in the experiment are as follows:

(1) $$\begin{array}{c} \text{accuracy}=\frac{\text{TP}+\text{TN}}{\text{TP}+\text{TN}+\text{FP}+\text{FN}},\\ \text{precision}=\frac{\text{TP}}{\text{TP}+\text{FP}},\\ \text{recall}=\frac{\text{TP}}{\text{TP}+\text{FN}},\\ \text{F}1=\frac{2*\text{TP}}{\text{N}+\text{TP}-\text{TN}}, \end{array}$$

where TP represents the number of samples whose positive sentiment polarity labels are correctly predicted as positive by the model. TN represents the number of samples whose negative sentiment polarity labels are correctly predicted by the model to be negative. FP represents the number of samples whose negative class sentiment polarity labels are mispredicted as positive by the model. FN represents the number of samples whose positive sentiment polarity labels are mispredicted as negative by the model. N represents the total sample size.

### 2.2. Analysis of Experimental Results

In order to analyze the classification performance of the model used in this study on the evaluation data, the selected comparison models are mainly SVM [19], k-nearest neighbor (KNN) [20], logistic regression (LR) [21], and decision tree (DT) [22]. The experimental results of each model on the Restaurant dataset are shown in Table 2 and Figure 2. The experimental results of each model on Laptop review datasets are shown in Table 3 and Figure 3.

It can be seen from the experimental results on the Restaurant dataset that the USVM used in this study has the best classification performance. The reasons are as follows: first, the experimental results on the four indicators are higher than those of other classifiers. Second, the accuracy and precision obtained based on USVM are similar in size, which shows that the algorithm used in this study has good performance for the classification of positive and negative samples. This is very important for imbalanced data.

From the experimental results on the Laptop dataset, it can be seen that the classification performance of the USVM used in this study is significantly better than other classifiers. The performance of traditional SVM is relatively poor, because the imbalanced data are constructed in this study, so the traditional SVM algorithm has a poor classification effect on this kind of data set. Among the other classifiers, the performance of DT is relatively stable, but it is slightly lower than USVM as a whole, so this study finally chooses USVM to classify the collected museum evaluation data.

## 3. Sentiment Analysis of Museum User Experience Evaluation Data

First, we used a *Python* crawler to get the museum user review text and store it as a CSV file. Second, data preprocessing is performed on the comment text, such as mechanical deduplication, cleaning, word segmentation, and word vector transformation. Third, the USVM is used to classify the data and obtain positive and negative text data. Finally, the semantic user satisfaction analysis of the comment text is carried out, and relevant conclusions and museum construction and maintenance strategies are drawn. The research framework is shown in Figure 4.

### 3.1. Data Acquisition and Preprocessing

The network questionnaire is mainly expanded from the aspects, as listed in Table 4. A total of 8,280 pieces of experience evaluation data of museum users were obtained through online surveys. Since there is a certain degree of noise in the texts crawled on the Internet, it is necessary to clean the collected comment texts to ensure more accurate analysis results. The comment text with less than 2 characters and duplicate content are deleted to ensure the availability and uniqueness of the comment text. After cleaning the comment text, a total of 8,000 valid comment texts were retained.

### 3.2. Sentiment Classification of Museum User Experience Data

Using the 10-fold cross-validation method, 6000 items in the dataset are used as the training set, and the remaining 2000 items are used as the test set to test the sentiment classification performance of the museum evaluation data. The number of categories is 3, which represent three emotions: satisfaction, neutrality, and dissatisfaction.  Table 5 lists examples of sentiment classification rule words.  Table 6 lists examples of manual labeling.

Considering that in the user experience evaluation data of the museum, the data of negative evaluation are much less than the number of positive and neutral evaluations. In view of this situation, the USVM used in this study is suitable for classifying data. The classification results based on USVM are listed in Table 7.

It can be seen from Table 7 that the accuracy of the training set and test set of the algorithm is greater than 86%, and the classification effect is ideal.

### 3.3. Interactive Service Comment Text Extraction and Analysis

#### 3.3.1. Interactive Comment Text Extraction

On the basis of the above classification, this part extracts comments under different sentiment classifications and sets the comments extracted from the “satisfied” text set as positive comments and the ones extracted from the “neutral” text set as neutral comments, and negative comments are extracted from the “unsatisfactory” text set. We analyze and summarize the feature words related to interactive reviews, as listed in Table 8

According to the constructed interactive comment vocabulary dictionary, each comment in the “satisfactory” comment text set, “neutral” comment text set, and “unsatisfactory” comment text set is traversed, respectively. This comment text sentence is then extracted. A total of 3200 related interactive evaluations were extracted. It can be seen from Table 9 that the positive description interaction accounts for 61% of the total comment text, which is 1952. Negative texts accounted for 21% or 672. Neutral texts accounted for 18% or 576.

#### 3.3.2. Recognition of Interactive Elements of User Attention Based on Word Frequency Method

This part uses the word frequency analysis method to analyze the word frequency of positive and negative logistics reviews. The “stutter” word segmentation tool of the *Python* language is used to segment the positive comment text and make word frequency statistics. The word frequency statistics are shown in Figure 5. In the top 10 word frequencies in Figure 5, 1 is convenient, 2 is clear, 3 is easy to use, 4 is interesting, 5 is smooth, 6 is rich, 7 is wonderful, 8 is novel, 9 is fast, and 10 is simple.

Based on the results shown in Figure 5, these are the factors that users pay more attention to in the museum experience process. Through word frequency statistics, it can be analyzed whether users pay more attention to whether the interaction is smooth and the operability is simple and clear.

Figure 6 shows a graph of the top 10 word frequency statistics of negative comment texts. Based on the results shown in Figure 6, it can be analyzed that users will generate negative comments due to the complex interactive interface and unclear feedback information. In the top 10 word frequencies in Figure 6, 1 is inconvenient, 2 is fuzzy, 3 is not easy to use, 4 is boring, 5 is laggy, 6 is monotonous, 7 is not exciting, 8 is not novel, 9 is too slow, and 10 is not fun.

#### 3.3.3. Apriori-Based Analysis of the Impact of Interactivity on User Experience Emotion

In order to further mine the relationship between the interaction-related elements in the comment text and the user experience emotion, this part uses the Apriori algorithm based on association rules to mine the relationship between the interactive comment words in the user comment text and the user experience emotion. Our purpose is to try to discover the interactivity-related vocabulary that affects user satisfaction and to further analyze the impact of interactivity on user experience emotions. Among them, the text data come from the “satisfied” and “dissatisfied” interactive comment texts extracted above. The words of user satisfaction and dissatisfaction come from the sentiment dictionary, as listed in Table 6.

Association rules can reflect the frequency of two itemsets appearing at the same time. The Apriori algorithm mainly generates association rules through the discovery of frequent itemsets [23, 24]. This part applies association rules to mine the co-occurrence of interaction-related words and satisfaction words in positive and negative comments. The metrics describing association rules include support (support) and confidence (confidence). When the support and confidence between itemsets are greater than the threshold, it is considered to have a strong association relationship. In the study, the support (A⟶B) represents the probability of word A and word B appearing at the same time, the confidence (A⟶B) indicates the probability that word A appears and word B also appears at the same time, and their expressions are as follows:

(2) $$\begin{array}{c} \text{support}\left(\text{A}\Rightarrow \text{B}\right)=P\left(A\cup B\right), \end{array}$$

(3) $$\begin{array}{c} \text{confidence}\left(\text{A}\Rightarrow \text{B}\right)=P\left(\frac{B}{A}\right)\frac{\text{support}\left(A\cup B\right)}{\text{support}\left(A\right)}. \end{array}$$

Lift (A⟶B) is used to reflect the correlation between vocabulary A and vocabulary B. If lift >1, then the occurrence of A and B is positively correlated. If lift <1, then the occurrence of A and B is negatively correlated. If lift = 1, then A and B are independent of each other, and the expression is as follows:

(4) $$\begin{array}{c} \text{lift}\left(\text{A}\Rightarrow \text{B}\right)=\frac{\text{confidence}\left(A\cup B\right)}{P\left(A\right)P\left(B\right)}. \end{array}$$

The study sets lift >1, support >0.01, and confidence > average as the threshold to mine the association between words.

In this section, we apply *R* language to segment and extract the comment text. The extracted words are replaced by synonyms, and words such as “extremely satisfied,” “ very satisfied,” and “satisfied” are replaced with “very satisfied” and “ok,” “okay,” and “good” are replaced with “good.” The related words such as smooth interaction and free operation are replaced with “good interaction” and converted into a transaction type data set for Apriori correlation analysis. The data processing results and visualization are listed in Table 9:

It can be seen from Table 9 that the words “easy to use,” “smooth,” “beautiful,” and “interesting” in the positive comments all have an effective correlation with the words “very satisfied” and “very good” that express satisfaction (lift >1). It can be seen that the interactive function of the birth digital museum positively affects the user's experience emotion, especially the interactive function represented by the above words has a high correlation with satisfaction.

According to the confidence value (confidence) value, the correlation analysis between words is mined as follows: {easy to use}⟶{satisfied} confidence is 0.7895, {convenient}⟶{easy to use} confidence is 0.6542, indicating that when the words “easy to use” and “convenient” appear, the probability of the word “easy to use” is more than 65%; {good ease of use}⟶{satisfied} confidence level is 0.6029, indicating that it is expected that the system is convenient to use and conforms to the usage habits of the system. The confidence level of {clear}⟶{very good} is 0.5321, and the confidence level of {good feedback}⟶{satisfied} is 0.5352, indicating that users have a high demand for picture clarity during the use of the entire museum system. The confidence level of {interesting}⟶{good entertainment} is 0.4434, the confidence level of {fun}⟶{good entertainment} is 0.3848, and the confidence level of {good entertainment}⟶{satisfied} is 0.4658, which indicates that entertainment is also very concerned. The confidence level of {fluency}⟶{good} is 0.4126, which indicates that users have certain requirements for the fluency and operability of the system. The confidence level of {wonderful}⟶{good visuality} is 0.2728, and the confidence level of {good visuality}⟶{satisfaction} is 0.5875, which indicates that users are very concerned about the visual experience presented by the system. The confidence level of {easy to operation}⟶{satisfied} is 0.4659, which indicates that users want the system to be simple and not too complicated.

The top 5 items sorted in descending order according to the lexical support value are as follows: {not stuck}⟶{good operability}, {fluency}⟶{good}, {clear feedback}⟶{good feedback}, {interesting}⟶{good entertainment}, and {wonderful}⟶{good visuality}. The support degree indicates the probability of word combinations appearing in all comments; at the same time, it also reflects the ranking of users' attention to a certain extent. Among them, similar words represented by “fluency” and “interesting” have the highest probability of appearing in positive comments.

After tokenizing the negative comment text, the arules package of the *R* language is used for association analysis. First, the extracted words are replaced with synonyms, words such as “click,” “input,” “check,” and “switch” are replaced with “interaction”, “not very good” and “too bad” with “dissatisfied,” and the “fuzzy” and “not clear” with “unclear”, the related words indicating inconvenient operation are replaced with “poor operability,” the comment words are converted into a transaction type data set, and Apriori correlation analysis is performed. The data processing results and visualization are listed in Table 10.

It can be seen from Table 10 that in the negative comments, the words that have an effective correlation with the satisfaction words are {not easy to use}⟶{too bad}, {poor picture}⟶{uninteresting}, and {monotonous}⟶{dislike}. It can be seen that the main factors causing the negative emotions of consumers are the fluency of the system and the unsatisfactory picture sense. The vocabulary combinations that are effectively related to words with poor operability are {stuck}⟶{dissatisfied}, {slow feedback}⟶{poor interaction}, and {cumbersome}⟶{poor operability}, and this result is similar to the correlation analysis result of positive comment text, which further indicates that the system interactivity elements are highly correlated with user satisfaction.

According to the confidence value, the correlation analysis results of words can be obtained as follows: (1) The confidence level of {not easy to use}⟶{too bad} is 0.5228; (2) The confidence level of {inconvenient}⟶{dissatisfied} is 0.4225; 3) The confidence level of {cumbersome}⟶{poor operability} is 0.4048. When the words “not easy to use” and “inconvenient” appear in the comments, there will be a 40% to 55% probability that words similar to “poor operability” will be mentioned. The confidence levels of {poor picture}⟶{uninteresting} and {monotonous}⟶{dislike} are 0.4866 and 0.3738, respectively, which indicates that users believe that the monotony of the picture will affect the user experience and thus reduce their satisfaction. The confidence levels of {stuck}⟶{dissatisfied} and {slow feedback}⟶{poor interaction} are 0.3994 and 0.5961, respectively, which indicates that users believe that interactivity is a major factor affecting their satisfaction.

According to the descending order of the vocabulary support value, the top 3 are {not easy to use}⟶{too bad}, {boring}⟶{dissatisfied}, and {stuck}⟶{dissatisfied}, and the corresponding support values are 0.0869, 0.0817, and 0.0731, respectively. Support indicates the proportion of word combinations appearing in all comments and also reflects the ranking of user attention to a certain extent. Among them, similar words represented by “not easy to use” and “stuck” have the highest probability of co-occurring in negative comments.

## 4. Conclusion

This study takes the user experience review texts of digital museums as the research object and proposes a USVM model that can deal with imbalanced data to classify related text sentiments. Based on the classification results, the top 10 word frequencies of different categories are extracted. The Apriori algorithm based on association rules is used to analyze the correlation between the different emotions of users and the interactive experience of digital museums. By analyzing the experimental results, we can find some problems existing in the construction and use of the existing digital museum and put forward corresponding improvement strategies accordingly. Conclusions are drawn from the above research: (1) the ease of use of digital museums is positively related to user satisfaction, that is, the simple and clear operation will help users to feel satisfied, while the cumbersome operation will easily lead to negative comments from users; (2) the interactive performance factors that museum users pay attention to when using the system are clear feedback, interactive entertainment, freedom of operation, consistent interactive vision, and easy and clear operation; (3) users' dissatisfaction with museum interactivity mainly focuses on unclear feedback, lack of interactivity, cumbersome operation, and inconsistent interaction. In this study, three-level classification is adopted for the processing of comment text sentiment, and it can be upgraded to five-level sentiment classification in the future, so as to dig deeper into the internal perception elements of users. At the same time, future research can enrich the data collection channels and indicators of concern and carry out comparative research on the mining of comment texts on different platforms or indicators.

## Figures and Tables

**Figure 1:** USVM algorithm flow chart.

**Figure 2:** Comparison of classification results on the Restaurant dataset.

**Figure 3:** Comparison of classification results on the Laptop dataset.

**Figure 4:** Sentiment analysis process.

**Figure 5:** Top 10 word frequency statistics of positive comment text.

**Figure 6:** Top 10 word frequency statistics of negative comment text.

**Algorithm 1:** A denoising algorithm.

**Algorithm 2:** An oversampling method.

**Algorithm 3:** An undersampling method.

**Table 1:** Experimental dataset.

Dataset	Positive		Neutral		Negative	
	Train	Test	Train	Test	Train	Test
Restaurant	2164	728	637	196	807	196
Laptop	994	341	464	169	870	128

**Table 2:** Experimental results on the Restaurant dataset.

Model	Accuracy	Precision	Recall	F1
SVM	0.7745	0.8215	0.8477	0.8344
KNN	0.8098	0.8531	0.8129	0.8325
LR	0.8956	0.8606	0.8533	0.8569
DT	0.8258	0.8366	0.8050	0.8205
USVM	0.8757	0.8664	0.8566	0.8615

**Table 3:** Experimental results on Laptop.

Model	Accuracy	Precision	Recall	F1
SVM	0.6716	0.7521	0.6988	0.7245
KNN	0.7342	0.7652	0.8012	0.7828
LR	0.7365	0.7788	0.7569	0.7677
DT	0.7869	0.7952	0.7763	0.7856
USVM	0.8038	0.8335	0.8532	0.8432

**Table 4:** Questionnaire survey evaluation indicators.

First indicator	Secondary indicators	First indicator	Secondary indicators
Evaluation of visual	Color matching	Evaluation of interactivity	Ease of use
	Typesetting		Clear feedback
	Illustration design		Interactive entertainment
	Navigation design		Freedom of operation
	Page layout		Interactive visual consistency
	Button shape		Simple and clear operation

Evaluation of the function	Display function	Evaluation of information content	Accuracy
	Comment function		Content validity
	Interactive function		Amount of information
	Research function		Emotional support
	Entertainment function		Relevance
	Education function		Value
	Collection function		

**Table 5:** Example of sentiment classification rule words.

Sentiment classification	Typical vocabulary examples
Satisfied	Very good, very satisfied, very satisfied, not bad, ok, very beautiful, very realistic, and magnificent
Neutral	a little, barely, not very, average, and mediocre
Dissatisfied	Not smooth, disappointed, dissatisfied, disliked, not flashy enough, inconvenient, lacking, inconsistent, and uninteresting

**Table 6:** Examples of manual marking.

Sentiment classification	Label	Text example
Satisfied	1	1. Wow, I really like it, it feels like being there. 2. The online high-definition big picture exhibition is great, and you can even see the clothes of the characters.
Neutral	0	1. Okay, at least you can visit the museums without going out. 2. Such a museum is generally interactive.
Dissatisfied	−1	1. Lack of interesting and vivid explanations, it is boring. 2. On the whole, I am a little disappointed, the 3D effect is not dazzling enough.

**Table 7:** Sentiment classification results of museum user experience evaluation.

Data set	Accuracy	Precision	Recall	F1
Training set	0.8973	0.8645	0.8965	0.8802
Test set	0.8606	0.8176	0.8256	0.8216

**Table 8:** Examples of interactive comment feature words.

Index	Feature word example
Ease of use	Convenient, troublesome, simple, difficult to use, and easy to use
Clear feedback	Clear, clear, blurry, too dark, and too bright
Interactive entertainment	Funny, funny, interesting, cute, boring, boring, and so funny
Freedom of operation	Smooth, not stuck at all, not stuck, very smooth, a little stuck, and not moving
Interactive visual consistency	Rich, wonderful, classic, novel, and good looking
Simple and clear operation	Simple, fast, and clear at a glance

**Table 9:** Analysis results of the correlation between positive reviews and satisfaction.

Rules	Lift	Support	Confidence
{Easy to use}⟶{satisfied}	6.5323	0.0112	0.7895
{convenient}⟶{easy to use}	5.2546	0.0108	0.6542
{Good ease of use}⟶{satisfied}	7.6440	0.0132	0.6029
{Clear}⟶{very good}	3.3865	0.0228	0.5321
{Clear feedback}⟶{good feedback}	4.5123	0.0420	0.4652
{Good feedback}⟶{satisfied}	1.9758	0.0136	0.5352
{interesting}⟶{good entertainment}	3.7549	0.0349	0.4434
{fun}⟶{good entertainment}	3.1718	0.0256	0.3848
{Good entertainment}⟶{satisfied}	2.2938	0.0243	0.4658
{fluency}⟶{good}	1.6284	0.0466	0.4126
{Not stuck}⟶{good operability}	2.0236	0.0501	0.3102
{wonderful}⟶{good visuality}	5.7431	0.0332	0.2728
{novel}⟶{satisfaction}	4.8313	0.0284	0.3006
{Good visuality}⟶{satisfaction}	5.7652	0.0119	0.5875
{easy}⟶{good}	1.3526	0.0132	0.7643
{Clear at a glance}⟶{easy to operate}	3.5435	0.0157	0.5456
{Easy to operate}⟶{satisfied}	6.0348	0.0265	0.4659

**Table 10:** Analysis results of the correlation between negative reviews and satisfaction.

Rules	Lift	Support	Confidence
{Not easy to use}⟶{too bad}	3.7821	0.0869	0.5228
{inconvenient}⟶{dissatisfied}	5.4655	0.0466	0.4225
{cumbersome}⟶{Poor operability}	2.8632	0.0298	0.4048
{Poor picture}⟶{uninteresting}	1.9874	0.0373	0.4866
{monotonous}⟶{dislike}	4.3245	0.0198	0.3738
{stuck}⟶{dissatisfied}	2.4315	0.0731	0.3994
{Will not use again}⟶{dissatisfied}	5.2832	0.0698	0.4687
{Slow feedback}⟶{poor interaction}	2.0437	0.0385	0.5961
{disappointed}⟶{dissatisfied}	4.7633	0.0279	0.7325
{boring}⟶{dissatisfied}	3.7656	0.0817	0.7193
{missing}⟶{dislike}	1.7855	0.0693	0.5532

## Data Availability

The datasets used in this paper is available at https://alt.qcri.org/semeval2014/task4/index.php?id=data-and-tools.
